The article "N6-methyladenosine induced miR-143-3p promotes the brain metastasis of lung cancer via regulation of VASH1" was retracted in 2023. Reasons: errors in the images; duplicated images; unreliable data.

# *N6*-methyladenosine induced miR-143-3p promotes the brain metastasis of lung cancer via regulation of VASH1

**DOI:** 10.1186/s12943-019-1108-x

**Published:** 2019-12-10

**Authors:** Hongsheng Wang, Qianqian Deng, Ziyan Lv, Yuyi Ling, Xue Hou, Zhuojia Chen, Xiaoxiao Dinglin, Shuxiang Ma, Delan Li, Yingmin Wu, Yanxi Peng, Hongbing Huang, Likun Chen

**Affiliations:** 1 Guangdong Key Laboratory of Chiral Molecule and Drug Discovery, School of Pharmaceutical Sciences, Sun Yat-sen University, Guangzhou, 510006 Guangdong China; 2 Department of Medical Oncology, State Key Laboratory of Oncology in South China, Collaborative Innovation Center for Cancer Medicine, Sun Yat-sen University Cancer Center, Guangzhou, 510060 Guangdong China; 3 Cancer Center, Sun Yat-Sen Memorial Hospital, Sun Yat-Sen University, Guangzhou, 510120 Guangdong China; 4 Department of Medical Oncology, Henan Cancer Hospital, the Affiliated Cancer Hospital of Zhengzhou University, 127 Dongming Road, Zhengzhou, 450008 Henan China; 5 Department of Medical Oncology, Zhongshan City People Hospital, Zhongshan, 528403 Guangdong China

**Keywords:** miR-143-3p, Brain metastasis, Lung cancer, VASH1, VEGFA, Tubulin

## Abstract

**Background:**

Brain metastasis (BM) is one of the principal causes of mortality for lung cancer patients. While the molecular events that govern BM of lung cancer remain frustrating cloudy.

**Methods:**

The miRNA expression profiles are checked in the paired human BM and primary lung cancer tissues. The effect of miR-143-3p on BM of lung cancer cells and its related mechanisms are investigated.

**Results:**

miR-143-3p is upregulated in the paired BM tissues as compared with that in primary cancer tissues. It can increase the invasion capability of in vitro blood brain barrier (BBB) model and angiogenesis of lung cancer by targeting the three binding sites of 3’UTR of vasohibin-1 (VASH1) to inhibit its expression. Mechanistically, VASH1 can increase the ubiquitylation of VEGFA to trigger the proteasome mediated degradation, further, it can endow the tubulin depolymerization through detyrosination to increase the cell motility. m^6^A methyltransferase Mettl3 can increase the splicing of precursor miR-143-3p to facilitate its biogenesis. Moreover, miR-143-3p/VASH1 axis acts as adverse prognosis factors for in vivo progression and overall survival (OS) rate of lung cancer.

**Conclusions:**

Our work implicates a causal role of the miR-143-3p/VASH1 axis in BM of lung cancers and suggests their critical roles in lung cancer pathogenesis.

## Introduction

Brain metastasis (BM), which occurs in 20–40% of advanced stage cancers, is one of the most common adult intracranial malignancies [1]. Clinical management of BM patients with cancer has limited control efficiency. The survival times after BM diagnosis of cancer patients remain poor and less than 12 months [2]. Lung cancer is the most common primary site for secondary BM [3]. Upon diagnosis, BM is identified in about 10% of all lung cancer patients [4]. It has been reported that about 40% of lung adenocarcinoma (LAD) patients end up with BM at some point during their illness [2]. BM is one of the principal causes of morbidity and mortality for lung cancer patients. The survival of lung cancer patients with BM is limited to mere weeks to few months upon administration of multimodal treatment [4]. So far, the molecular events that govern metastatic development of lung cancer remain frustrating cloudy.

The article "N6-methyladenosine induced miR-143-3p promotes the brain metastasis of lung cancer via regulation of VASH1" was retracted in 2023. Reasons: errors in the images; duplicated images; unreliable data.

Accumulating data have indicated that microRNAs (miRNAs), one type of small non-coding RNAs of 18–25 nt, can inhibit translation and/or negatively regulate stability of mRNAs by binding to the 3′-untranslated region (3′-UTR) of targets to act as either tumor oncogenes or suppressors depending on the target mRNAs [5]. miRNAs play an important role in progression and metastasis of lung cancers [6]. For example, miRNAs have important roles in gefitinib-induced apoptosis and epithelial-mesenchymal transition (EMT) of non-small cell lung cancer (NSCLC) cells in vitro and in vivo [7]. miR-224/−520c-dependent TUSC3 deficiency enhances the metastatic potential of NSCLC cells through alteration of three unfolded protein response pathways [8]. Few studies indicated that intracellular and exosome miRNAs can regulate the BM [9, 10]. To date, miRNAs involved in lung cancer BM have been rarely characterized.

In this study, we aimed to identify miRNAs that regulate the BM of lung cancers by analysing differentially expressed miRNAs from paired lung primary and BM cancer tissues. We found a set of miRNAs were altered in BM tissues as compared to the primary cancers, which, spearheaded by miR-143-3p, converged on and repressed the expression of vasohibin-1 (VASH1). VASH1 has been primarily found to be the first endothelial cells (ECs)-intrinsic factor that has an inhibitory effect on angiogenesis [11]. Recently, VASHs were identified as the first tubulin-detyrosinating enzymes, a cell-autonomous role in regulating the cytoskeleton [12–14]. We reported here that miR-143-3p overexpression, or VASH1 silencing, fosters metastatic propensities of lung cancer cells, enhances their angiogenic capabilities, and endows tubulin depolymerization. Further, m^6^A methylation induced cleavage of precursor miRNA is responsible for the upregulation of miR-143-3p in BM tissues. Our work implicated a causal role for the miR-143-3p/VASH1 axis in BM of lung cancers and suggested their critical roles in lung cancer pathogenesis.

The article "N6-methyladenosine induced miR-143-3p promotes the brain metastasis of lung cancer via regulation of VASH1" was retracted in 2023. Reasons: errors in the images; duplicated images; unreliable data.

## Materials and methods

### Patient sample collection

Additional file 1: Table S1 and Additional file 1: Table S2 (Additional file 1) contain the detailed information of two cohorts of patients analysed in the current study. All tissue samples were histologically confirmed lung cancer with or without BM. Samples were collected from the Cancer Center of Sun Yat-sen University between January 2012 and February 2014. Lung cancer tissues and paired fresh brain metastases were acquired from patients with BMs undergoing surgery. Brain metastasis tissues were adequately dissected from surrounding stromal tissues. The tissue samples of cohort 1 were selected by an experienced pathologist immediately after surgical resection, snapped frozen in liquid nitrogen, and stored at − 80 °C for further RNA extraction. The tissue samples of cohort 2 were paraffin-embedded for section. For all of the patients who participated in this study, written consent forms approved by the Ethical Committee of Sun Yat-sen University according to the Chinese Ethical Regulations were signed and documented. Clinical data were reviewed retrospectively from medical records.

### Database (DB) analysis

The expression of miR-143-3p and VASH1 in lung cancer was analyzed by use of Kaplan-Meier plotter (http://kmplot.com/analysis/), a comprehensive online platform which can assess the effect of 54,675 genes on survival based on 10,293 cancer samples [15]. The expression of VASH1 in lung cancer patients was analyzed by use of data obtained from the Oncomine Database (www.oncomine.org) as follows: Selamat Lung, Talbot, Su and Landi. The sample information and expression data were available in the Gene Expression Omnibus (GEO) database [Accession nos. GSE32863 (Selamat Lung), GSE1775 (Talbot Lung), GSE7670 (Su Lung), and GSE10072 (Landi Lung) at www.ncbi.nlm.nih.gov/geo].

The correlations between expression of VASH1 and overall survival rate of lung cancer patients were analyzed by use of LinkedOmics (http://www.linkedomics.org), which is a publicly available portal that includes multi-omics data from all of 32 cancer types from The Cancer Genome Atlas (TCGA) project. The LinkedOmics web allowed flexible exploration of associations between a molecular or clinical attribute of interest and all other attributes, providing the opportunity to analyze and visualize associations between billions of attribute pairs for each cancer cohort [16].

### Experimental animals and xenograft models

BALB/c nude mice (4 weeks old) were purchased from Sun Yat-sen University Animal Center (Guangzhou, China) and raised under pathogen-free conditions. All animal experiments complied with Zhongshan School of Medicine Policy on Care and Use of Laboratory Animals. For subcutaneous transplanted model, control and miR-143-3p stable A549 cells (5 × 10^6^ per mouse, *n* = 5 for each group) were diluted in 200 μL PBS + 200 μL Matrigel (BD Biosciences) and subcutaneously injected into immunodeficient mice to investigate tumor growth. When tumor volume in each group reached approximately 100 mm^3^, mice were sacrificed, and tumors were removed and weighted for use in histology and further studies. The tumor volume was calculated using the formula V = 1/2× larger diameter × (smaller diameter) ^2^.

The article "N6-methyladenosine induced miR-143-3p promotes the brain metastasis of lung cancer via regulation of VASH1" was retracted in 2023. Reasons: errors in the images; duplicated images; unreliable data.

For in vivo lung colonization model, mice were injected with control or miR-143-3p stable A549 cells (1 × 10^6^ per mouse, *n* = 5 for each group) via tail vein to analyse the lung colonization. Eight weeks after injection, mice were sacrificed and colonized lung tumors were analyzed.

To investigate whether miR-143-3p/VASH1 axis can regulate the in vivo BM of lung cancer cells, control, miR-143-3p stable over expression (o/e), VASH1 stable o/e, and miR-143-3p/VASH1 dual stable o/e A549 cells resuspended in 100 μL PBS were injected into the right ventricle of nude mice (1 × 10^6^ per mouse, *n* = 8 for each group) according to previous studies [17, 18]. The animals were killed 8 weeks later. Incidence of brain metastasis was quantified on the basis of histology.

### Statistical analyses

Data were reported as mean ± standard deviation (SD) from at least three independent experiments unless otherwise specified. Values for capillary tube formation and luciferase activity assays were from three independent experiments. Data were analyzed by two-tailed unpaired Student’s t-test between two groups and by One-Way ANOVA followed by Bonferroni test for multiple comparisons. Statistical analyses were carried out using SPSS 16.0 for Windows. A *p*-value of < 0.05 was considered to be statistically significant. *p < 0.05, **p < 0.01; NS, no significant.

## Results

### miR-143-3p is correlated with the BM and progression of lung cancer

To identify potential miRNAs involved in the BM of lung cancer, we analysed miRNA expression profiles in 6 matched pairs of primary lung cancer and BM tissues by use of the mercury LNA™ microRNA Array. There were 20 miRNAs upregulated and 4 miRNAs down regulated in BM tissues as compared to that in primary tissues with the folds greater than 2 (Fig. 1a). Among the upregulated miRNAs, only miR-27b, miR-143-3p, and miR-145 were upregulated in each BM tissue as compared to that in the matched primary lung cancer tissues (Additional file 1: Figure S1A, B, C). We then checked the expression of miR-27b, miR-143-3p, miR-145, and miR-192 in primary lung cancer tissues with (*n* = 10) or without (*n* = 10) BM by in situ hybridization (ISH). The results showed that only miR-143-3p was significantly increased in BM positive lung cancer patients as compared to that in negative patients (Fig. 1b). Dimitrova et al. [19] suggested that expression of miR-143/145 in the tumor stroma promotes lung tumorigenesis. Results of ISH showed that miR-143-3p can be detected in both stroma and tumor cells in lung cancer tissues with or without BM, while the levels of miR-143-3p in tumor cells were greater than that in stroma cells (Additional file 1: Figure S1D). All these results suggested an intrinsic increase in the expression of miR-143-3p in metastatic lung cancer cells and tissue.

The article "N6-methyladenosine induced miR-143-3p promotes the brain metastasis of lung cancer via regulation of VASH1" was retracted in 2023. Reasons: errors in the images; duplicated images; unreliable data.

**Fig. 1:** miR-143-3p is correlated with the BM and progression of lung cancer. **a** The miRNA expression profiles in 6 matched pairs of primary lung cancer and BM tissues were analysed by use of the mercury LNA™ microRNA Array. The miRNAs with variation fold greater than 2 were showed. **b** The expression of miR-27b, miR-143-3p, miR-145, and miR-192 in lung cancer patients with (*n* = 10) or without (*n* = 10) BM was checked by in situ hybridization (ISH). **c** The expression of carcinoembryonic antigen (CEA) in miR-143-3p + (*n* = 38) or miR-143-3p- (*n* = 28) lung cancer patients. **d** The diameter of tumor in miR-143-3p + (*n* = 38) or miR-143-3p- (*n* = 28) lung cancer patients when diagnosis. **e** Kaplan-Meier survival curves of OS based on miR-143-3p expression in lung cancer patients (data from online bioinformatics tool Kaplan-Meier plotter). The log-rank test was used to compare differences between the two groups. **f** Kaplan-Meier survival curves of OS based on miR-143-3p expression in lung cancer patients (data from TCGA database). The log-rank test was used to compare differences between the two groups. Scale bar = 200 μm

We therefore checked the association between miR-143-3p and progression of lung cancer. The 66 lung cancer patients were divided into miR-143-3p positive (+, *n* = 38) and negative (−, *n* = 28) group according to the results of ISH (Additional file 1: Table S2). Our data showed that the expression of miR-143-3p in BM+ (25/34) was significantly (*p* < 0.01, χ^2^ test) greater than that in BM- (13/32) lung cancer patients. Further, miR-143-3p + lung cancer patients showed significant (*p* < 0.05, *t* test) greater levels of carcinoembryonic antigen (CEA, Fig. 1c) and tumor diameter at diagnosis (Fig. 1d) than that of miR-143-3p- patients. It implies an increasing tendency of miR-143-3p expression during malignant transformation of lung cancer. No significant difference had been observed for the gender, age, or T/N stage of lung cancer patients (Additional file 1: Table S2 and Additional file 1: Figure S1E). Using the online bioinformatics tool Kaplan-Meier plotter [20] (Fig. 1e) and data from TCGA data base (Fig. 1f), we found that lung cancer patients with increased levels of miR-143-3p showed reduced overall survival (OS). It indicated that miR-143-3p is correlated with the BM and progression of lung cancer.

The article "N6-methyladenosine induced miR-143-3p promotes the brain metastasis of lung cancer via regulation of VASH1" was retracted in 2023. Reasons: errors in the images; duplicated images; unreliable data.

#### miR-143-3p triggers EMT, invasion of BBB model, and angiogenesis of lung cancer

We then evaluated the potential functions of the identified miRNAs on the progression of lung cancer. We transfected A549 cells with miR-27b, miR-143-3p, miR-145, and miR-192 constructs (Additional file 1: Figure S2A). Wound healing assay showed that miR-143-3p had the greatest capability to promote the in vitro migration of A549 cells among all measured miRNAs (Fig. 2a, Additional file 1: Figure S2B). qRT-PCR showed that the expression of miR-143-3p was upregulated in lung cancer cells as compared with that in human bronchial epithelial cells (HBEC), while the expression of miR-143-3p in endothelial cells such as HBMEC, HUVEC and PAEC cells were comparable or slightly greater than that in lung cancer cells (Fig. 2b). Among the measured lung cancer cells, H1299 had the highest, while H1975 had the lowest, levels of miR-143-3p (Fig. 2b). Over expression of miR-143-3p also triggered the wound closure of H1975 cells (Additional file 1: Figure S2C). In vitro transwell assay confirmed that miR-143-3p can trigger the invasion of both A549 and H1975 cells (Fig. 2c). Further, over expression of miR-143-3p in A549 cells lost their cobblestone-like epithelial morphology and assumed a spindle-like fibroblast appearance, while inhibitor of miR-143-3p showed inverse morphology variation (Additional file 1: Figure S2D). We further evaluated the expression of cell migration and EMT related biomarkers in cells transfected with or without miR-143-3p. The data showed that miR-143-3p can decrease the expression of E-Cad, while increase the expression of FN, Vim, MMP2, and MMP-9 in A549 cells (Fig. 2d). We further established the in vitro blood brain barrier (BBB) model by use of human brain microvascular endothelial cells (HBMEC, Fig. 2e) according to the previous study [21]. Our data showed that miR-143-3p can increase the invasiveness through in vitro BBB model of both A549 and H1975 cells (Fig. 2f). These results suggested that over expression of miR-143-3p can increase the dissemination and invasiveness through in vitro BBB model of lung cancer cells.

The article "N6-methyladenosine induced miR-143-3p promotes the brain metastasis of lung cancer via regulation of VASH1" was retracted in 2023. Reasons: errors in the images; duplicated images; unreliable data.

**Fig. 2:** miR-143-3p triggers EMT, invasion of BBB model, and angiogenesis of lung cancer cells. **a** The quantitative results of wound healing assay of A549 cells transfected with miRNAs for 48 h. **b** The relative expression of miR-143-3p in lung cancer cell A549, H1975, H292, H1650 and H1299 cells, human bronchial epithelial cells (HBEC), HBMEC, HUVEC, and pulmonary artery endothelial cells (PAEC) was checked by qRT-PCR. **c** Cells were transfected with scramble RNA (Con) or miRNA-143 for 24 h, the cell invasion was measured by use of transwell assay and quantitatively analyzed. **d** A549 cells were transfected with control or miR-143-3p for 48 h, the expression of cell motility markers was measured by western blot analysis (*left*) and quantitatively analyzed (*right*). **e** The in vitro models of BBB. HBMECs grown on a Transwell membrane. **f** A549 or H1975 cells transfected with or without miR-143-3p were allowed to invade the in vitro BBB model for 48 h. The invaded cells were measured (*left*) and quantitatively analyzed (*right*). **g** Tube formation was evaluated in HUVECs cultured for 12 h in medium collected from A549 or H1975 cells transfected with or without miR-143-3p. The tube formation was recorded (*left*) and quantitatively analyzed (*right*). **h** After transfected with or without miR-143-3p for 24 h, the expression of VEGFA in lung cancer cells was measured by western blot analysis (*left*) and quantitatively analyzed (*right*). **i** H1299 cells transfected with or without miR-143-3p inhibitor were allowed to invade the in vitro BBB model for 48 h. The invaded cells were measured (*left*) and quantitatively analyzed (*right*). **j** Tube formation was evaluated in HUVECs cultured for 12 h in medium collected from H1299 cells transfected with or without miR-143-3p inhibitor. The tube formation was recorded (*left*) and quantitatively analyzed (*right*). **k** After transfected with or without miR-143-3p inhibitor for 24 h, the expression of VEGFA in H1299 cancer cells was measured by western blot analysis (*left*) and quantitatively analyzed (*right*). Data are presented as the mean ± SD from three independent experiments. *p < 0.05, ** *p* < 0.01 compared with control. Scale bar = 100 μm

We then investigated the roles of miR-143-3p on the proliferation of lung cancer cells. Results showed that miR-143-3p had no effect on the proliferation of either A549 or H1975 cells after transfected for 24 h (Additional file 1: Figure S2E). Over expression of miR-143-3p can slightly but not significantly decrease the proliferation of A549 after treated for 3 days (Additional file 1: Figure S2F). Clone formation assay showed that over expression or inhibitor of miR-143-3p had no effect on the colonization of A549 cells (Additional file 1: Figure S2G). These data suggested that miR-143-3p had limited effect on the proliferation and colonization of lung cancer cells.

The article "N6-methyladenosine induced miR-143-3p promotes the brain metastasis of lung cancer via regulation of VASH1" was retracted in 2023. Reasons: errors in the images; duplicated images; unreliable data.

We further checked the potential roles of miR-143-3p in angiogenesis of lung cancer cells by tube formation assay since neo-angiogenesis is a hallmark of cancer BM [22]. Results showed that the condition medium of A549 and H1975 cells transfected with miR-143-3p significantly promoted the tube formation of HUVECs (Fig. 2g). Further, over expression of miR-143-3p can increase the expression of VEGFA in lung cancer cells including A549, H1975, H292 and H1650 (Fig. 2h). These results suggested that miR-143-3p can increase the angiogenesis and expression of VEGFA in lung cancer cells.

We then checked the potential roles of miR-143-3p inhibitor on the invasion of in vitro BBB model and angiogenesis of H1299 cells since it had the highest level of miR-143-3p (Fig. 2b). Our data showed that inhibitor of miR-143-3p can significantly decrease the in vitro invasiveness through BBB model of H1299 cells (Fig. 2i). Consistently, transfection of miR-143-3p inhibitor can inhibit tube formation of HUVECs (Fig. 2j) and expression of VEGFA in H1299 cells (Fig. 2k). It further confirmed the promotion roles of miR-143-3p on the progression of lung cancer.

#### VASH1 mediates miR-143-3p induced cell dissemination and angiogenesis

The potential targets of miR-143-3p were predicted by combinatorial use of five different web-based databases (miRanda, miRDB, miRwalk, RNA22, and TargetScan). Among the 25 identified targets from 5 databases (Additional file 1: Table S3), we checked the mRNA expression of cancer metastasis or angiogenesis related genes including VASH1 [12], USP54 [23], WASF3 [24], GABRB3 [25], IGFBP5 [26], and HK2 [27] in cells transfected with miR-143-3p. Over expression of miR-143-3p decreased the expression of VASH1, while not others, in both A549 (Fig. 3a) and H1975 (Fig. 3b) cells. miR-143-3p can also decrease the expression of WASF3 in A549 cells (Fig. 3a). Considering that the down regulation of WASF3 can suppress the cancer progression [24], we further investigated the potential roles of VASH1 in miR-143-3p induced progression of lung cancer. Consistently, over expression of miR-143-3p can also decrease the mRNA expression of VASH1 in H292, H1650, and H1299 cells (Additional file 1: Figure S3A). Western blot analysis confirmed that over expression of miR-143-3p can decrease the expression of VASH1 in all measured lung cancer cells (Fig. 3c). Consistently, miR-143-3p inhibitor can increase the expression of VASH1 in both A549 and H1975 cells (Additional file 1: Figure S3B). The relative expression of miR-143-3p was negatively corelated with that of VASH1 in all measured lung cancer and HBEC cells (Fig. 3d). The data showed that miR-143-3p can negatively regulate the expression of VASH1.

The article "N6-methyladenosine induced miR-143-3p promotes the brain metastasis of lung cancer via regulation of VASH1" was retracted in 2023. Reasons: errors in the images; duplicated images; unreliable data.

**Fig. 3:** VASH1 mediates miR-143-3p induced cell dissemination and angiogenesis. **a** & **b** A549 (A) or H1975 (**b**) cells were transfected with control or miR-143-3p for 24 h, the mRNA expression of potential targets was measured by qRT-PCR. **c** Lung cancer cells were transfected with control or miR-143-3p for 24 h, the expression of VASH1 was measured by western blot analysis (*left*) and quantitatively analyzed (*right*). **d** The relative expression of miR-143-3p and mRNA of VASH1 was negative correlated in measured lung cancer and HBEC cells. **e** Schematic representation of three positions of miR-143-3p binding with the 3’UTR of VASH1 mRNA. **f** A549 cells were co-transfected with control, miR-143-3p, pmiR-GLO-WT, and pmiR-GLO-Mut-a/b/c for 24 h, the value of firefly luciferase (F-luc) was normalized to that of the Renilla luciferase (R-luc). **g**-**i** A549 cells were co-transfected with control, miR-143-3p, vector, or VASH1 construct for 48 h, (**g**) the expression of FN and E-Cad was measured by measured by western blot analysis (*left*) and quantitatively analyzed (*right*); **h** The invasion of BBB model for 48 h was measured (*left*) and quantitatively analyzed (*right*); **i** The tube formation was evaluated in HUVECs cultured for 12 h (*left*) and quantitatively analyzed (*right*). Data are presented as the mean ± SD from three independent experiments. *p < 0.05, ** *p* < 0.01 compared with control, NS, no significant. Scale bar = 100 μm

We further investigated whether miR-143-3p can directly target the mRNA of VASH1. Three potential binding sites have been observed in the 3’UTR of VASH1 (Fig. 3e). We cloned the wild type 3’UTR of VASH1 to generate pmiR-GLO-WT andmutated the three potential binding sites (UCAUCUC to U**A**A**CA**U**U**), respectively, to generate pmiR-GLO-Mut-a/b/c. As expected, luciferase assay showed that over expression of miR-143-3p can significantly decrease the wild-type reporter activity, however, all three mutants can rescue the miR-143-3p induced down regulation of luciferase activity with the capability in the order of Mut-a > Mut-b > Mut-c (Fig. 3f). In H1299 cells, miR-143-3p inhibitor can increase the wild-type reporter activity, while the three mutants can rescue the miR-143-3p induced up regulation of luciferase activity (Additional file 1: Figure S3C). Collectively, these results indicated that VASH1 is a direct target of miR-143-3p in lung cancer cells with the site “a” as the most important site for the binding of miR-143-3p.

The article "N6-methyladenosine induced miR-143-3p promotes the brain metastasis of lung cancer via regulation of VASH1" was retracted in 2023. Reasons: errors in the images; duplicated images; unreliable data.

We further evaluated whether VASH1 was involved in miR-143-3p regulated cell dissemination and angiogenesis. Wound healing assay showed that over expression of VASH1 can significantly rescue miR-143-3p induced migration of A549 cells (Additional file 1: Figure S3D). Western blot analysis showed miR-143-3p induced down regulation of E-Cad and upregulation of FN was attenuated by over expression of VASH1 (Fig. 3g). In vitro BBB model confirmed that over expression of VASH1 can significantly rescue miR-143-3p increased invasiveness through in vitro BBB model of A549 cells (Fig. 3h). Further, condition medium of A549 transfected with VASH1 can significantly attenuate miR-143-3p induced the tube formation of HUVECs (Fig. 3i). These results indicated that VASH1 was involved in miR143 promoted dissemination and angiogenesis of lung cancer cells.

#### VASH1 mediates miR-143-3p induced angiogenesis via destabilization of VEGFA

VASH1 exhibits a feedback anti-angiogenic activity via induction by VEGF though unclear mechanisms [28, 29]. In lung cancer cells, over expression of VASH1 can decrease the expression of VEGFA in both A549 and H1975 cells tested by western blot analysis (Fig. 4a) or ELISA (Additional file 1: Figure S4A). Further, overexpression of VASH1 can attenuate miR-143-3p induced upregulation of VEGFA in both A549 (Fig. 4b) and H1975 (Additional file 1: Figure S4B) cells. Although the promotion roles of VEGFA in angiogenesis have been well illustrated [30], we further investigated whether VEGFA is involved in miR-143-3p regulated angiogenesis of lung cancer by treating HUVEC cells with or without recombinant VEGFA (rVEGFA). Our data showed that rVEGFA can increase the tube formation of HUVECs and further rescue VASH1 suppressed tube formation (Fig. 4c). It indicated that VASH1 was involved in miR-143 regulated expression of VEGFA and angiogenesis of lung cancer.

**Fig. 4:** VASH1 mediates miR-143-3p induced angiogenesis via destabilization of VEGFA. **a** A549 or H1975 cells were transfected with vector control or VASH1 construct for 24 h, the expression of VEGFA was measured by western blot analysis (*left*) and quantitatively analyzed (*right*). **b** A549 control or miR-143-3p stable cells were transfected with vector control or VASH1 construct for 24 h, the expression of VEGFA was measure by western blot analysis (*left*) and quantitatively analyzed (*right*). **c** Tube formation was evaluated in HUVECs cultured for 12 h in medium collected from A549 cells transfected with vector or pcDNA/VASH1 and supplemented with or without 10 ng/ml rVEGFA. **d** A549 cells were transfected with control, miR-143-3p, vector control or VASH1 construct for 24 h, the mRNA expression of VEGFA was measured by qRT-PCR. **e** Analysis of VEGFA mRNA in non-ribosome portion (<40S), 40S, 60S, 80S, and polysome in A549 cells transfected with vector control or VASH1 constructs for 24 h. **f** A549 cells transfected with vector control or VASH1 constructs for 24 h were further treated with 10 μg/ml CHX for the indicated time periods. The expression of VEGFA was detected by western blot analysis (*left*) and quantitatively analyzed (*right*). **g** A549 cells transfected with vector control or VASH1 constructs for 24 h were further treated with 10 μg/ml CHX or 10 μM MG-132 for 6 h, the expression of VEGFA was detected by western blot analysis (*left*) and quantitatively analyzed (*right*). **h** A549 cells transfected with vector control or VASH1 constructs for 24 h in the presence of MG-132. After VEGFA was immunoprecipitated, the ubiquitination of VEGFA was examined by western blot analysis. An equal amount of VEGFA was loaded after IP according to a pre-Western blot. Data are presented as the mean ± SD from three independent experiments. *p < 0.05, ** *p* < 0.01 compared with control, NS, no significant. Scale bar = 100 μm

The mechanisms responsible for VASH1-inhibited VEGFA were further investigated. Our data showed that neither VASH1 nor miR-143-3p can influence the mRNA expression of VEGFA in A549 cells (Fig. 4d). Further, over expression of VASH1 had no effect on the mRNA stability of VEGFA (Additional file 1: Figure S4C). It indicated that VASH1 regulated expression of VEGFA is due to the post-transcriptional regulation. We further performed linear sucrose gradient fractionation to assess the association between polyribosomes and VEGFA mRNA to investigate whether VASH1 can regulate the mRNA translation of VEGFA. As shown in Fig. 4e, over expression of VASH1 had no significant effect on the distribution of VEGFA mRNA in both fractions containing translation-dormant complexes and translating polyribosomes, which is indicative of no translation variation. Thus, reduction of VEGFA by VASH1 seems to occur at the post-translational level rather than the regulation of its translation.

The article "N6-methyladenosine induced miR-143-3p promotes the brain metastasis of lung cancer via regulation of VASH1" was retracted in 2023. Reasons: errors in the images; duplicated images; unreliable data.

We then investigated whether VASH1 can directly interact with VEGFA to influence its expression. Co-IP showed that VASH1 can not bind with VEGFA in A549 cells (Additional file 1: Figure S4D). Protein stability assay showed that VASH1 can decrease the half-life of VEGFA in A549 cells (Fig. 4f). The half-lives of VEGFA in A549 cells transfected with or without VASH1 were 8.1 and 2.9 h, respectively. To further confirm that VASH1 post-translationally suppressed the expression of VEGFA, A549 cells transfected with or without VASH1 were further treated with MG132 to inhibit proteasome activity or CHX to block translation. The data showed that MG-132 can attenuate the VASH1 suppressed VEGFA expression in A549 cells, while CHX had no similar effect (Fig. 4g). Since ubiquitylation is critical for proteasome mediated protein degradation, we hypothesized that VASH1 may modify ubiquitylation of VEGFA. Immunoprecipitation results showed that ubiquitylation of VEGFA was dramatically increased in VASH1-transfected A549 cells (Fig. 4h). It indicated that VASH1 can increase the ubiquitylation mediated proteasome degradation of VEGFA in lung cancer cells. These data suggested that VASH1 mediated miR-143-3p induced angiogenesis via destabilization of VEGFA protein.

#### VASH1 mediates miR-143-3p induced depolymerization of microtube

Recently, VASH1 has been demonstrated to encode tubulin detyrosinating activity [12–14]. The reversible tyrosination/detyrosination of α-tubulin is critical for the stability and dynamicity of microtube (MTs) and important for invasion of cancer cells [14]. Firstly, over expression of miR-143-3p can decrease the levels of detyrosinated tubulin (deY-Tub) in A549 cells (Fig. 5a). Consistently, inhibitor of miR-143-3p can increase the levels of deY-Tub in H1299 cells (Additional file 1: Figure S5A). Further, over expression of VASH1 can abolish miR-143-3p decreased deY-Tub in A549 cells (Fig. 5a). Neither miR-143-3p nor VASH1 can influence the protein expression of total α-tubulin (Fig. 5a). Confocal results showed that the expression of VASH1 was decreased in miR-143-3p over expression cells, however, the VASH1 colocalized with MTs in both control and miR-143-3p over expression cells (Fig. 5b).

**Fig. 5:** VASH1 mediates miR-143-3p induced depolymerization of microtube. **a** A549 cells were transfected with control, miR-143-3p, vector or VASH1 construct for 24 h, the expression of deY-Tub and tubulin was measured by western blot analysis (*left*) and quantitatively analyzed (*right*). **b** The expression and localization of α-tubulin (*red*) and VASH1 (*green*) in control and miR-143-3p stable A549 cells were checked by confocal. **c** The expression and localization of α-tubulin (*red*) and deY-Tub (*green*) in control and miR-143-3p stable A549 cells were checked by confocal. **d** The control and miR-143-3p stable A549 cells were treated with or without PTX (2 μM) for 2 h, the expression of deY-Tub was measured by western blot analysis (*left*) and quantitatively analyzed (*right*). **e** The control and miR-143-3p stable A549 cells were treated with or without PTX (2 μM) for 2 h, the invasion of BBB model for 24 h was recorded (*left*) and quantitatively analyzed (*right*). **f** Immunofluorescence staining of microtubule re-growth of control and miR-143-3p stable A549 cells transfected with or without VASH1 construct after treatment with nocodazole (50 μM) for 10 min, followed by a washout and incubation in fresh culture medium at 37 °C for 10, 30, or 120 min. **g** Control and miR-143-3p stable A549 cells transfected with or without VASH1 construct after treatment with nocodazole (50 μM) for 10 min, followed by a washout and incubation in fresh culture medium at 37 °C for 10, 30, or 120 min. The levels of deY-tub and total tubulin were measured by western blot analysis (*left*) and quantitatively analyzed (*right*). **h** A549 cells were transfected with control, miR-143-3p, vector or VASH1-C169A- construct for 24 h, the expression of deY-Tub and tubulin was measured by western blot analysis (*left*) and quantitatively analyzed (*right*). **i** The control and miR-143-3p stable A549 cells were transfected with vector or VASH1-C169A construct for 24 h, the invasion of in vitro BBB model was recorded (*left*) and quantitatively analyzed (*right*). **j** A549 cells were transfected with vector control or VASH1-C169A construct for 24 h, the protein expression was recorded (*left*) and quantitatively analyzed (*right*). Data are presented as the mean ± SD from three independent experiments. *p < 0.05, ** *p* < 0.01 compared with control. Red scale bar = 100 μm. White scale bar = 10 μm

Having identified miR-143-3p can regulate the detyrosination of α-tubulin via regulation of VASH1, we next determined whether it could affect the polymerized microtubule population. We stained A549 cells using antibodies against α-tubulin and deY-Tub. The signal for deY-Tub colocalized with MMTs in wild-type cells, further, the expression of deY-Tub decreased in miR-143-3p over expression cells (Fig. 5c).

The article "N6-methyladenosine induced miR-143-3p promotes the brain metastasis of lung cancer via regulation of VASH1" was retracted in 2023. Reasons: errors in the images; duplicated images; unreliable data.

To substantiate whether deY-Tub was involved in miR-143-3p regulated migration of lung cancer cells, we treated cells with paclitaxel (PTX), which can lead to a robust increase in α-tubulin detyrosination in various cells [12]. Consistently, PTX can blunt miR-143-3p suppressed expression of deY-Tub in A549 cells (Fig. 5d). Further, both wound healing assay (Additional file 1: Figure S5B) and in vitro BBB model (Fig. 5e) showed that PTX can significantly attenuate miR-143-3p triggered migration and invasion capability of BBB model of A549 cells, respectively. It suggested that VASH1 induced α-tubulin detyrosination was involved in miR-143-3p triggered dissemination and BM of lung cancer cells.

Alpha-tubulin acetylation or detyrosination classically marks stable MTs [14]. To investigate whether the association of VASH1 with MTs influences their dynamic properties, we treated A549 cells with nocodazole and monitored MT re-growth after nocodazole washout. Polymerized MT fibers in control cells were evident already 10 min after the washout, however, MT fibers were detected only 120 min after nocodazole washout in miR-143-3p stable cells (Fig. 5f). The over expression of VASH1 can fast the polymerization and attenuate miR-143-3p delayed polymerization of MTs (Fig. 5f). Western blot analysis confirmed that the expression of deY-Tub in miR-143-3p stable cells were delayed as compared with that in control cells, while over expression of VASH1 can attenuate this delay effect (Fig. 5g). Next, we analyzed the effect of miR-143-3p on MT depolymerization by treating control or miR-143-3p stable cells with increasing concentrations of nocodazole. In control cells, MTs began to partially depolymerize at 5-μM concentrations (with some MT fibers still detectable), and total depolymerization was achieved with 10 μM nocodazole. While 1 μM nocodazole induced partially depolymerization of MT fibers in miR-143-3p stable cells. Further, 5 μM nocodazole was sufficient to induce complete depolymerization (Additional file 1: Figure S5C). Furthermore, treatment with 1 μM nocodazole did not change the level of deY-Tub in control cells while decreased the level of deY-Tub in miR-143-3p expressing cells (Additional file 1: Figure S5D). This suggested that miR-143-3p can regulate the deY-Tub to influence the polymerization of MTs via a VASH1 dependent manner.

To confirm that VASH1 mediated detyrosination of α-tubulin was involved in miR-143-3p induced reprogramming of MTs and cell dissemination, we generated VASH1 mutant VASH1-Cys169Ala, which has been proved to be essential for VASH-dependent induction of deY-Tub [12]. Our data showed that VASH1-C169A failed to rescue miR-143-3p decreased deY-Tub of A549 cells (Fig. 5h). Further, over expression of VASH1-C169A failed to attenuate the miR-143-3p destabilized the MT network (Fig. 5f) and miR-143-3p triggered invasion of in vitro BBB model (Fig. 5i). In addition, VASH1-C169A had no significant effect on the expression of E-Cad and FN of A549 cells (Fig. 5j) or cell migration (Additional file 1: Figure S5E). These results confirmed that VASH1 mediates miR-143-3p induced reprogramming of MTs via its tubulin detyrosinating activity.

#### The m^6^A modification regulates the expression of miR-143-3p in lung cancer cells

The potential mechanisms responsible for the upregulation of miR-143-3p in lung cancer and BM tissues were investigated. Firstly, treatment with 5-aza-dC (a DNA methyltransferase inhibitor) had no significant effect on miR-143-3p expression in either A549 or H1975 cells (Additional file 1: Figure S6A), suggesting that DNA methylation might not be involved in miR-143-3p expression in lung cancer cells. The role of histone acetylation in miR-143-3p expression was investigated by treating A549 cells with specific inhibitors of HDAC1, 3, 4, 6 and 8 or broad-spectrum HDAC inhibitors such as SAHA and NaB (Additional file 1: Figure S6B). The data showed that these HDAC inhibitors had no significant effect on miR-143-3p expression in A549 cells (Additional file 1: Figure S6B). These data suggested that DNA methylation or histone acetylation might not be responsible for the upregulation of miR-143-3p in lung cancer cells.

The article "N6-methyladenosine induced miR-143-3p promotes the brain metastasis of lung cancer via regulation of VASH1" was retracted in 2023. Reasons: errors in the images; duplicated images; unreliable data.

It has been reported that *N6*-methyladenosine (m^6^A) modification can regulate the biogenesis of miRNAs [31, 32]. We found that knockdown the expression of Mettl3, the key m^6^A methyltransferase (“writer”) in mammalian cells [33], can decrease the expression of miR-143-3p in both A549 and H1975 cells (Fig. 6a, and Additional file 1: Figure S6C). We further knocked down the expression of Mettl3 in A549 cells by two siRNAs (Additional file 1: Figure S6D). Our data showed that both two siRNAs for Mettl3 can also significantly decrease the expression of miR-143-3p in A549 cells (Additional file 1: Figure S6E). Consistently, over expression of Mettl3 can increase the expression of miR-143-3p in both A549 and H1975 cells (Fig. 6b, and Additional file 1: Figure S6F). Intriguingly, sh-Mettl3 significantly increased the expression of precursor-miR-143-3p in A549 and H1975 cells (Fig. 6c). However, sh-Mettl3 had no effect on the distribution of precursor-miR-143-3p between cytoplasm and nucleus in A549 cells (Fig. 6d). In addition, sh-Mettl3 had no significant effect on promoter activity of miR-143-3p (Additional file 1: Figure S6G) or the expression of primary miR-143-3p (Additional file 1: Figure S6H), suggesting that m^6^A had no effect on the transcription of miR-143-3p.

**Fig. 6:** The m^6^A regulates the expression of miR-143-3p in lung cancer cells. **a** Cells were transfected with si-NC or si-Mettl3 for 24 h, the expression of miR-143-3p was checked by qRT-PCR. **b** Cells were transfected with vector control or Mettl3 constructs for 24 h, the expression of miR-143-3p was checked by qRT-PCR. **c** A549 cells were transfected with sh-Control or sh-Mettl3 for 24 h, the expression of precursor miR-143-3p was measured by qRT-PCR. **d** A549 cells were transfected with (sh-Control) or sh-Mettl3 for 24 h, the expression of precursor miR-143-3p in cytoplasm and nucleus was measured by qRT-PCR. **e** & **f** A549 cells were transfected with sh-Control or sh-Mettl3 for 24 h and further treated with Act-D for the indicated times, and mature and precursor miR-143-3p expression was measured by qRT-PCR. **g** m^6^A RIP-qPCR analysis of precursor and mature miR-143-3p in A549 cells. **h** A549 cells were transfected with si-NC or si-Dicer for 24 h, the expression of Dicer was measured by western blot analysis. **i** A549 cells were transfected with vector control, Mettl3 construct, si-NC or si-Dicer alone or together for 24 h, the expression of mature miR-143-3p was measured by qRT-PCR. Data are presented as the mean ± SD from three independent experiments. *p < 0.05, **p < 0.01 compared with control

The results that sh-Mettl3 can decrease the mature-miR-143-3p while increase precursor-miR-143-3p indicated that m^6^A may regulate the splicing of precursor miRNA. This was confirmed that sh-Mettl3 had no effect on the half-life of mature-miR-143-3p (Fig. 6e) while significantly increased the half-life of precursor of miR-143-3p (Fig. 6f) in A549 cells. Further, m^6^A RNA-immunoprecipitation (RIP) qPCR showed there was significant enrichment of precursor miR-143-3p, while not mature miR-143-3p, in m^6^A antibody levels as compared to that in IgG (Fig. 6g). To further confirm that m^6^A modification can trigger the generation of miR-143-3p via accelerating the splicing the precursor miRNA, we knocked down the expression of Dicer (Fig. 6h), which cleaves pre-miRNA into short single-stranded miRNA [34]. Our data showed that the knockdown of Dicer abolished Mettl3 induced upregulation of miR-143-3p in A549 cells (Fig. 6i). The results indicated that m^6^A can facilitate the splicing of precursor miR-143-3p to generate mature miRNA in lung cancer cells.

The article "N6-methyladenosine induced miR-143-3p promotes the brain metastasis of lung cancer via regulation of VASH1" was retracted in 2023. Reasons: errors in the images; duplicated images; unreliable data.

#### The miR-143-3p/VASH axis and in vivo BM of lung cancer

At this point, we asked whether there was a link between m^6^A methylation-regulated miR-143-3p/VASH1 axis and BM of lung cancer by use of three animal cohorts. Firstly, both control and miR-143-3p stable A549 cells were injected subcutaneously into nude mice. Mice were sacrificed when the tumor volumes were about 100 mm^3^ for each group. IHC results showed that miR-143-3p can decrease the expression of VASH1 and deY-tub, while increase the expression of CD31, a biomarker for microvessel density in tumor tissues, in xenografts as compared with that in the control group (Fig. 7a). Further, over expression of miR-143-3p can increase the expression of FN, and vim in xenograft tumor tissues (Fig. 7a). It suggested that over expression of miR-143-3p can increase the in vivo potential of metastasis and angiogenesis of lung cancer when the tumor volumes were comparable.

**Fig. 7:** The miR-143-3p/VASH axis and in vivo BM of lung cancer. **a** The expression of VASH1, deY-tubulin, CD31, FN, and Vim in control and miR-143-3p groups were measured by IHC (*left*) and quantitatively analyzed (*right*). **b** & **c** The control and miR-143-3p A549 cells were injected into the nude mice by tail vein injection. Representative images of metastatic lung tumors and the H&E staining results were shown (*left*), and the number of lung tumors were quantitatively analyzed (*right*). **d** Metastasis was detected by histology; BM (100 X) and BM (200 X). **e** Percentage of BM in all measured groups. **f** Expression of VASH1 in NSCLC (cancer) and adjacent normal tissues from Oncomine dataset (Selamat). **g** VASH1 expression in lung cancers of T1 (*n* = 145), T2 (*n* = 182), and T3 (*n* = 35) stages from TCGA database. **h** Kaplan-Meier survival curves of OS based on VASH1 mRNA expression in lung cancer patients. The log-rank test was used to compare differences between two groups. **i** The IHC scores of VASH1 in BM+ (*n* = 34) or BM- (*n* = 32) lung cancer patients. **j** The IHC scores of VASH1 in miR-143-3p+ (*n* = 38) or miR-143-3p- (*n* = 28) lung cancer patients. (K) Kaplan-Meier survival curves of OS of miR-143-3p^−^VASH1^high^ and miR-143-3p^+^VASH1^low^ group of lung cancer patients. The log-rank test was used to compare differences between two groups. Data are presented as the mean ± SD from three independent experiments. *p < 0.05, **p < 0.01 compared with control. Scale bar = 100 μm

To further determine the impacts of miR-143-3p on in vivo progression of lung cancer, both control and miR-143-3p stable A549 cells were injected into the BALB/c nude mice, respectively, by tail vein injection to analyze lung colonization. Eight weeks after injection, experiment was terminated and lungs were analyzed to report the presence of metastatic tumors. As shown in Fig. 7b & c, the number of lung tumors derived from miR-143-3p A549 cells was significantly increased compared to control cells, suggesting that over expression of miR-143-3p increased the lung colonization of lung cancer cells in vivo.

To investigate whether miR-143-3p/VASH1 axis can regulate the in vivo BM of lung cancer cells, A549 control, miR-143-3p stable over expression (o/e), VASH1 stable o/e, and miR-143-3p/VASH1 dual stable o/e cells were injected into the right ventricle of nude mice [17]. One mouse died 1 week after intracardiac injection with the miR-143-3p o/e cells, and this mouse was excluded from the study. In the A549-Mock group, one mouse died at the 7th wk. after intracardiac injection. However, histological examination confirmed that BM had not occurred in this mouse, and therefore, we included it in the final analysis. Consequently, there were 8 mice in the A549-Mock group and 7 mice in the miR-143-3p o/e group at the time of the final analysis in the 7th wk. Histopathological analysis showed that the percentage of BM in the control group (3/8, 37.5%) was significantly lower than that in the miR-143-3p group (5/7, 71.1%). The percentage of BM in VASH1 o/e and miR-143-3p/VASH1 dual o/e was 12.5% (1/8) and 25.0% (2/8), respectively. It indicated that the miR-143-3p induced BM was abolished in the present of VASH1 (Fig. 7d and e). These data suggested that miR-143-3p/VASH1 was involved in the in vivo BM of lung cancer.

The article "N6-methyladenosine induced miR-143-3p promotes the brain metastasis of lung cancer via regulation of VASH1" was retracted in 2023. Reasons: errors in the images; duplicated images; unreliable data.

Since our data showed that increased expression of miR-143-3p showed reduced OS and increased BM, we further questioned the roles of VASH1 in lung cancer development. Decreased expression of VASH1 in cancer tissues than that in normal tissues was observed in all analyzed sets of data from Oncomine including Talbot (Additional file 1: Figure S7A), Su (Additional file 1: Figure S7B), Landi (Additional file 1: Figure S7C), and Selamat (Fig. 7f) lung samples. Significant reduced expression levels of VASH1 from T1 to T3 stage of lung cancer tissues were also observed (Fig. 7g), implying a decreasing tendency of VASH1 expression during malignant transformation. Consistently, diminishing expression levels of VASH1 from N0 to N2 stage of lung cancer tissues were observed (Additional file 1: Figure S7D). Using the online bioinformatics tool Kaplan-Meier plotter [20] (Fig. 7h), we found that lung cancer patients with decreased expression of VASH1 showed reduced OS.

We further checked whether VASH1 was involved in miR-143-3p induced BM of our cohort 2 lung cancer patients. The expression of VASH1 in 66 lung cancer patients (BM+ 34 cases, BM- 32 cases) was checked by IHC. The data showed that the expression of VASH1 in BM+ group was significantly lower than that in BM- group of lung cancer patients (Fig. 7i). Consistently, the expression of VASH1 in miR-143-3p + group was significantly lower than that in miR-143-3p- group of lung cancer patients (Fig. 7j). The patients in our cohort were separated to miR-143-3p^−^VASH1^high^ and miR-143-3p^+^VASH1^low^ group, the data showed that the lung cancer patients of miR-143-3p^+^VASH1^low^ had significant reduced OS compared to that of miR-143-3p^−^VASH1^high^ patients (Fig. 7k). These results suggested that the miR-143-3p/VASH1 axis triggers the in vivo progression and BM of lung cancer.

## Discussion

In the present study, we identified the expression of miR-143-3p was increased in BM as compared to the primary lung cancer tissues and correlated with the progression of lung cancer. Gain and loss of function studies revealed that miR-143-3p can increase the invasion capability of in vitro BBB model and angiogenesis of lung cancer cells by targeting the three binding sites of 3’UTR of VASH1 to inhibit its expression. Mechanistically, VASH1 can increase the ubiquitylation of VEGFA to trigger its degradation, further, it can endow the tubulin depolymerization though detyrosination. m^6^A methyltransferase Mettl3 can facilitate miR-143-3p biogenesis via promoting its cleavage from precursor to mature miRNA. In vivo data confirmed the essential role of VASH1 in miR-143-3p induced BM of lung cancer. As summarized in Fig. 8, m^6^A-induced miR-143-3p can promote the BM of lung cancer via VASH1 mediated reprograming angiogenesis and MTs depolymerization.

The article "N6-methyladenosine induced miR-143-3p promotes the brain metastasis of lung cancer via regulation of VASH1" was retracted in 2023. Reasons: errors in the images; duplicated images; unreliable data.

**Fig. 8:** Model of the m^6^A-induced miR-143-3p promotes the BM of lung cancer via regulation of angiogenesis and microtubules though VASH1

Our study revealed that miR-143-3p is upregulated in BM tissues, further, it can trigger the invasion of in vitro BBB model and angiogenesis of lung cancer. Consistently, the recent study found that stromal expression of miR-143/145 can promote the neoangiogenesis of lung cancer [19]. The first large-scale miRNA in situ NSCLC tissue hybridization analysis found significantly increased expression of miR-143 in tumor cells and adjoining stromal cells in comparison to non-malignant tissues [35]. Similarly, the relative expression of miR-143 was higher in glioblastoma (GBM) patients compared to that in control ones [36]. Endogenous miR-143 can trigger the intestinal epithelial regeneration, pulmonary fibrosis, and skin wound healing [26]. Further, miR-143 can induce EMT and modulate the expression of junction proteins of cells derived from STAT3C/NeuT transgenic mice mammary tumors [37]. However, miR-143 has also been characterized as tumor suppressors in colorectal [38], breast [39] and bladder [40] cancer. In addition, it has been reported that miR-143 can suppress the proliferation and migration of lung cancer NCI-H23 cells via targeting LIM Domain Kinase 1 (Limk1) [41]. Differences in the cancers, cell types and tumor heterogeneity could contribute to these divergent results [42]. It also might be due to that miR-143 has the tight temporal regulation effects on lung cancer progression, which favors extravasation while impairs fitness in the colonized tissue.

We found that VASH1 was involved in miR-143 triggered angiogenesis of lung cancers. The expression of HK2, which was previously reported to be the target of miR-143-3p [43], was not variated in lung cancer cells transfected with miR-143-3p. It indicated that the effect of miR-143 on HK2 expression might be cell line or cancer dependent. miR-143 was highly expressed in smooth muscle cells (SMCs) to modulate the angiogenic and vessel stabilization properties of endothelial cells (ECs) [44]. Mice with genetic deficiency of miR-143 exhibited reduced vascular tone and blood pressure control [45, 46]. Some preliminary studies indicated that VASH1 exhibits antitumor effects by inhibiting angiogenesis [47, 48], while knockdown of VASH1 is a crucial driver of tumor angiogenesis and metastasis [49]. VASH1 has been primarily found to be the first ECs-intrinsic factor to inhibit the angiogenesis with an unillustrated negative feedback mechanism [11, 29]. Herein we found for the first time that VASH1 can negatively regulate the expression of VEGFA via triggering its ubiquitylation and proteasome mediated degradation, which was evidenced by the results that VASH1 can decrease the half-life of VEGFA while had no effect on its mRNA expression. The results enrich our knowledge about the post-translational modifications (PTMs) and degradation of VEGFA, while the mechanisms responsible for VASH1 induced ubiquitylation of VEGFA need further studies.

miR-143-3p can reprogram the polymerization of MTs via the tubulin-detyrosinating activity of VASH1 in lung cancer cells. The cyclic removal and ligation of the C-terminal tyrosine of α-tubulin is one of the most important PTMs of unstable MTs and implicated in cellular processes such as mitosis and cell migration [14, 50]. While deY-Tub was characterized as very stable and long-lived MTs [51]. Our present study showed for the first time that the tubulin-detyrosinating activity of VASH1 is involved in miR-143-3p-induced invasion of in vitro BBB model of lung cancer cells, suggesting that the less stable MTs might be essential for BM of cancer cells. Consistently, the expression of tubulin tyrosine ligases such as TTLL12, which increases the tyrosinated tubulin and leads to disassembly of MTs, were markedly increased as the prostate cancer progresses from a benign to a metastatic stage [52]. While the stabilization of MTs by deletion of RCCD1 can attenuate the TGF-β-induced EMT process of NSCLC cells [53].

The article "N6-methyladenosine induced miR-143-3p promotes the brain metastasis of lung cancer via regulation of VASH1" was retracted in 2023. Reasons: errors in the images; duplicated images; unreliable data.

Finally, we explored whether m^6^A methylation, but not DNA methylation or histone acetylation, was involved in the upregulation of miR-143-3p in lung cancer cells. Mettl3 can trigger the splicing of precursor miR-143-3p to generate mature miR-143-3p, which was evidenced by knockdown of Dicer can abolish m6A regulated expression of miR-143. Few studies indicated that m^6^A can regulate the biogenesis of miRNAs through reduction of the binding of DGCR8 to pri-miRNAs [31, 32]. Alternatively, our present study found for the first time that m^6^A positively regulated the cleavage of precursor miRNAs. Considering that knowledge of the mechanism of RNA methylation is still in its infancy, additional discoveries of regulatory patterns mediated by m^6^A on the biogenesis and functions of miRNAs are worth verifying in the future.

In conclusion, we identified that miR-143-3p was involved in the BM of lung cancer cell via down regulation of VASH1. Moreover, we demonstrated novel mechanisms for VASH1 suppressed the expression of VEGFA, revealed that the tubulin-detyrosinating activity of VASH1 was essential for BM of lung cancer cells, and found that m^6^A can trigger the cleave of precursor miRNAs. Our results provided a potent target that may serve as a predictive marker of metastasis and an effective target for anti-metastatic therapies for lung cancer patients.

## Supplementary information

**Additional file 1: Figure S1.** miR-143-3p is correlated with the BM and progression of lung cancer. **Figure S2.** The effects of miRNAs on the malignancy of lung cancer cells. **Figure S3.** VASH1 mediates miR143 induced cell dissemination and angiogenesis. **Figure S4.** VASH1 mediates miR-143-3p induced angiogenesis via destabilization of VEGFA. **Figure S5.** VASH1 mediates miR-143-3p induced reprogramming of microtubules. **Figure S6**. m6A regulates the expression of miR-143-3p in lung cancer cells. **Figure S7.** The miR-143-3p/VASH axis and in vivo BM of lung cancer. **Table S1.** Clinical characteristics of 6 lung cancer patients with BM. **Table S2.** Clinical characteristics of lung cancer patients with or without BM. **Table S3.** The potential targets of miR-143-3p predicted by five different web-based databases.

## Data Availability

The detailed procedures of methods, seven figures and four tables are attached.

## Abbreviations

3’UTR: 3′-untranslated region
Act-D: Actinomycin D
BBB: Blood brain barrier
BM: Brain metastases
CHX: Cycloheximide
deY-Tub: detyrosinated tubulin
ECs: Endothelial cells
EMT: Epithelial-mesenchymal transition
GBM: Glioblastoma
HBEC: Human bronchial epithelial cells
HBMEC: Human brain microvascular endothelial cells
HUVECs: Human umbilical vein endothelial cells
IHC: Immunohistochemistry
ISH: In situ hybridization
LAD: Lung adenocarcinoma
miRNAs, m6A: N^6^-methyladenosine; microRNAs
MTs: Microtubes
NSCLC: Non-small cell lung cancer
OS: Overall survival
PTMs: Post-translational modifications
SD: Standard deviation
SMCs: Smooth muscle cells
TCGA: The cancer genome atlas
VASH1: Vasohibin-1
